# Post grafting time significantly influences royal jelly yield and content of macro and trace elements

This article has been retracted.

**DOI:** 10.1371/journal.pone.0238751

**Published:** 2020-09-08

**Authors:** Saad N. Al-Kahtani, El-Kazafy A. Taha

**Affiliations:** 1 Arid Land Agriculture Department, College of Agricultural Sciences and Foods, King Faisal University, Al-Ahsa, Saudi Arabia; 2 Economic Entomology Department, Faculty of Agriculture, Kafrelsheikh University, Kafrelsheikh, Egypt; Harran University, TURKEY

## Abstract

Royal jelly (RJ) is commercially harvested after the 4^th^ day of queen larval age. In the current study, it was harvested after 24, 48, 72, and 96 hours after grafting of 1-day larval age queens to investigate changes in macro and trace elements associated with harvesting time. The RJ yields were significantly affected by harvest time, and the highest yield was obtained 72 hours after grafting. The highest phosphorus (P) and zinc (Zn) contents were obtained from RJ harvested 24 hours after grafting. Royal jelly harvested 48 hours after grafting had the highest concentrations of magnesium (Mg), calcium (Ca), potassium (K), sodium (Na), iron (Fe), and manganese (Mn). Likewise, RJ harvested 96 hours after grafting had higher concentrations of copper (Cu). Royal jelly harvested 72 hours after grafting showed the second rank for P, Mg, Ca, K, Na, Fe, Cu, and Mn concentrations. In descending order, P, Mg, Ca, and K were the most dominant elements in RJ harvested at different times after grafting. The Mg, Ca, K, Na, Cu, and Mn concentrations in RJ were all positively correlated, and P, Fe, and Zn were positively correlated. The P and Zn were negatively correlated with Ca, Cu, and Mn. It was concluded that macro and trace element contents in RJ can differ depending on the harvest time after grafting. We recommend harvesting RJ at 72 hours after grafting for possible use as healthy nutritional human food supplement.

## Introduction

Royal jelly (RJ) is a valuable bee product released by the hypopharyngeal and mandibular glands located in the heads of worker honeybees. These glands become more active by the time the workers reach an age of 5–15 days [1–3]. Royal jelly is the diet of young honeybee larvae and plays the main role in caste differentiation of honeybees. The queen larvae receive RJ for 5 days, while the worker larvae receive RJ only for 3 days, and then receive a mixture of honey, pollen and water for 2 days. Thereafter, a queen of honeybee lives for several years, and the worker bees lives for a few months [4].

Royal jelly is a milky substance composed of proteins, sugars, lipids, vitamins, and individual elements [5–9]. It can be harvested in relatively small quantities from normally built queen cells [10], or commercially in comparatively larger amounts by using an artificial queen-rearing method [11–15].

The elements content in RJ have determined as ash [5, 6, 8, 9, 16–22]. The standard amount of ash in RJ is reportedly approximately 0.8–3% [23]. The element concentration of RJ produced in Saudi Arabia ranges from 2.16% in RJ harvested 24 hours after grafting to 3.03% in RJ harvested 72 hours after grafting [8]. However, the elements content in RJ produced have differed affected by the botanical and geographical origins and other biological factors related to the worker bees [24, 25].

Royal jelly is an important functional food parameter that possesses several health-promoting characteristics. It has been widely used in commercial healthy foods and medical products in many countries. Royal jelly has been approved to possess several functional properties such as antioxidant, antibacterial, antihypercholesterolemic, anti-inflammatory, antitumor, disinfectant, vasodilative and hypotensive activities [18, 26]. In addition, it has used to supplement many diseases, including cardiovascular, diabetes, cancer and Alzheimer’s disease [26]. The daily requirements of the individual elements in human nutrition have determined as 800–1200 mg P, 800 mg K, 800–900 mg Ca, 300–400 mg Mg, 6–22 mg Zn, 10–20 mg Fe, 4–5 mg Mn and 1–3 mg Cu [27, 28]. Trace elements play a vital role in the biomedical activities of RJ, as these have a variety of biological functions [18].

The nutritional and therapeutic characteristics of RJ have led to its inclusion in an increasing number of food products [7, 9, 18, 29–34]. Royal jelly is commercially harvested at the end of the 4^th^ day of queen larval age [2, 8, 35], but there are few reports on the element content of RJ harvested before this time. In the present study the effects of harvesting time on the macro and trace element contents of RJ were investigated, with a particular focus on elements that are essential for human nutrition [phosphorus (P), potassium (K), sodium (Na), magnesium (Mg), calcium (Ca), iron (Fe), zinc (Zn), copper (Cu), and manganese (Mn)].

## Materials and methods

### Royal jelly sampling

The RJ used in the study was produced at the apiary of the Training and Research Station, King Faisal University, Al-Ahsa (25°25′46″N, 49°37′19″E; 121 m above sea level), Saudi Arabia during February and March in 2019. One colony of the hybrid Carniolan honeybee (*Apis mellifera carnica* Pollmann) was selected as a breeder colony to provide all larvae used for grafting. Ten colonies of 10 frames each were selected for RJ production. Fifty wax cups were grafted with larvae that were 24 hours of age, and the cups were introduced into each colony. Royal jelly was harvested from the accepted queen cell cups 24, 48, 72, and 96 hours after grafting in previously weighed small bottles. The bottles with RJ were weighed using an electronic balance. The mean yield of RJ (mg/queen cell) for every harvest time was calculated by subtraction [8].

### Macro and trace elements extraction and analysis

Wet digestion with nitric acid [36] was used for element extraction. One gram of RJ from each harvest was digested in a Kjeldahl flask with 10 ml of 75% nitric acid (HNO_3_) for the oxidation of carbonaceous matter. The contents of the flask were heated 100–120 ºC, to evaporate the acid. Drops of perchloric acid (HClO_4_) were added until all the organic matter was oxidized. This point was reached when no further darkening of the solution occurred on continuous heating and a clear solution was obtained. It was cooled and gauged to 50 ml with distilled water. A blank experiment was carried out by adding the same amount of nitric acid to 1 ml distilled water. An atomic absorption spectrophotometer (Avanta E, GBC, Australia) was used to detect calcium (Ca), copper (Cu), iron (Fe), magnesium (Mg), manganese (Mn), potassium (K), sodium (Na) and zinc (Zn). A UV-VIS spectrophotometer (UV-2550 Shimadzu, Kyoto, Japan) was used to detect the phosphorus (P) concentrations.

### Statistical analysis

The difference between harvesting times was tested by one-way analysis of variance (ANOVA), which indicated significant difference for harvesting times. The normality in data was tested by Shapiro-Wilk normality test, which indicated data were normally distributed. Therefore, the analyses were performed on original data. The ANOVA and Pearson’s correlational coefficients were used to assess differences and associations between the elements investigated via the PROC GLM function in SAS version 9.1 [37]. Duncan’s [38] multiple range test was used to compare means.

## Results

Royal jelly yields were significantly (*p* < 0.01) affected by harvest time (Table 1). The highest yield (318.5 mg/queen cell) was obtained 72 hours after grafting. The lowest yield (70.4 mg/queen cell) was obtained 24 hours after grafting (Fig 1).

**Fig 1:** Effect of harvesting time on royal jelly yield (mg/queen cell).

**Table 1:** Analysis of variance of yield and nutrient concentration in royal jelly.

Variable	SS	MS	F value	P value
RJ yield	125893.4	41964.5	1523.2	< 0.0001*
P	6198224.3	2066074.7	679959.0	< 0.0001*
Mg	32852748.7	10950916.2	2879108.0	< 0.0001*
Ca	7045039.8	2348346.6	697253.0	< 0.0001*
K	882608.6	294202.8	77788.1	< 0.0001*
Na	1212430.9	404143.6	150918.0	< 0.0001*
Fe	1876.9	625.6	312.8	< 0.0001*
Zn	6788.3	2262.7	1216.2	< 0.0001*
Cu	121.2	40.4	35.7	< 0.0001*
Mn	6.7	2.2	1393.5	< 0.0001*

Source of variation = post-grafting time, degree of freedom = 4, SS = sum of squares, MS = mean squares, * = significant.

The mean concentrations (mg/kg) of P (8636.7–10113.3), Mg (6920.5–9545.2), Ca (2806.2–4334.5), K (1630.0–4334.5), Na (193.0–675.0), Fe (43.4–76.3), Zn (32.8–78.7), Cu (34.4–39.9) and Mn (0.5–1.9) differed significantly (*p* < 0.01) at different harvesting times (Table 1). Royal jelly harvested 48 hours after grafting had the highest mean contents (mg/kg) of Mg (9545.2), Ca (4334.5), K (2126.2), Na (675.0), Fe (76.3) and Mn (1.9). The highest concentrations of P (10113.3) and Zn (78.7) were obtained from RJ harvested 24 hours after grafting. Royal jelly harvested 96 hours after grafting had higher concentrations of Cu (39.9). The lowest concentrations of Mg (6920.5), Ca (2806.2), K (1630.3), Na (193.2), Cu (34.4) and Mn (0.5) were present in RJ harvested 24 hours after grafting, and the lowest concentrations of P (8636.7), Fe (52.4), and Zn (32.8) were present in RJ harvested 96 hours after grafting (Table 2).

**Table 2:** Effects of different harvesting times on concentrations (mg/kg) of macro and trace elements in royal jelly.

Element	Time (hours) after grafting				Mean
	24	48	72	96	
**Macro elements**					
P	10113.3 ± 2.3^a^	9222.4 ± 1.8^c^	9245.3 ± 1.7^b^	8636.7 ± 1.4^d^	9304.4
Mg	6920.5 ± 1.8^d^	9545.2 ± 2.4^a^	9166.7 ± 1.7^b^	7053.3 ± 1.6^c^	8171.4
Ca	2806.2 ± 2.1^d^	4334.5 ± 1.4^a^	3652.4 ± 1.8^b^	3544.7 ± 1.5^c^	3584.5
K	1630.3 ± 2.2^d^	2126.2 ± 2.2^a^	1980.4 ± 1.3^b^	1750.2 ± 1.8^c^	1871.8
Na	193.2 ± 2.0^d^	675.1 ± 1.5^a^	640.0 ± 1.4^b^	205.3 ± 1.5^c^	428.4
**Trace elements**					
Fe	72.3 ± 1.4^b^	76.3 ± 1.7^a^	73.4 ± 1.3^b^	52 4 ± 1.2^c^	74.0
Zn	78.7 ± 1.6^a^	55.1 ± 1.5^b^	41.8 ± 1.2^c^	32.8 ± 0.9^d^	52.1
Cu	34.4 ± 1.3^b^	39.5 ± 1.0^a^	39.1 ± 0.4^a^	39.9 ± 1.2^a^	38.2
Mn	0.5 ± 0.0^c^	1.9 ± 0.1^a^	1.6 ± 0.0^a^	1.1 ± 0.0^b^	1.3

The values shown are means ± standard deviation. The means of each row followed by a different letter differed significantly.

There were relative abundances of P (46.3, 35.4, 37.3, and 40.5% of the total elements quantified), Mg (31.7, 36.6, 36.9, 64`and 33.1%), Ca (12.8, 16.6, 14.7 and 16.6%), K (7.5, 8.2, 8.0 and 8.2%) and Na (0.9, 2.6, 2.6, and 1.0%) for RJ harvested 24, 48, 72 and 96 hours after grafting, respectively (Table 3).

**Table 3:** Relative abundance (%) of macro elements in royal jelly at different harvesting times.

Elements	Time (hrs) after grafting				Average
	24	48	72	96	
P	46.3	35.4	37.2	40.5	39.8
Mg	31.7	36.6	36.9	33.1	34.6
Ca	12.8	16.6	14.7	16.6	15.2
K	7.5	8.2	8.0	8.2	8.0
Na	0.9	2.6	2.6	1.0	1.7

Concentrations of Mg, Ca, K, Na, Cu, and Mn in RJ were positively correlated (*r* = 0.54–0.98, *p* < 0.01) (Table 4). Concentrations of P, Fe, and Zn were positively correlated (*r* = 0.61–0.95, *P* < 0.01). Fe was positively correlated with K (*r* = 0.47, *p* < 0.05) and Mg (*r* = 0.61, *p* < 0.01). P and Zn were negatively correlated with Ca, Cu, and Mn (*r* = -0.51 to -0.85, *p* < 0.01).

**Table 4:** Pearson’s correlation coefficients for macro and trace elements in royal jelly.

	P	Mg	Ca	K	Na	Fe	Zn	Cu	Mn
P	1								
Mg	-0.24								
Ca	-0.61**	0.83**							
K	-0.40*	0.97**	0.94**						
Na	-0.22	0.99**	0.80**	0.96**					
Fe	0.61**	0.61**	0.19	0.47*	0.62**				
Zn	0.95**	-0.27	-0.51**	-0.37	-0.27	0.73**			
Cu	-0.85**	0.55**	0.75**	0.65**	0.54**	-0.41*	-0.81**		
Mn	-0.56**	0.93**	0.95**	0.98**	0.92**	-0.12	-0.54**	0.78**	1

*p < 0.05 (two-tailed)

**p < 0.01 (two-tailed).

## Discussion

All larvae used for grafting in the current study were obtained from the same queen, and reared for RJ production under the same colony conditions, so differences between the amounts of RJ/queen cell can reasonably be summarized to be due to differences in harvesting times [8]. Royal jelly yields in queen cells were related to the amounts of RJ required by each larval instar, which increases with larval age. The amount of RJ in a queen cell initially increased gradually with larva age, then it peaks on the 4^th^ day of larval age, then it decreased on the 5^th^ day of larval age. In commercial systems RJ is harvested on the 4^th^ day of larval age because that is when the yields are maximal [2, 8, 12, 14, 35].

In the current study, all RJ samples were produced in the same colonies, and all larvae used for grafting were derived from the same queen, so the observed differences in concentrations of macro and trace elements can reasonably be summarized to be due to the type of RJ introduced to the larvae at the different larval instars. There were numerous significant differences in element concentrations in RJ harvested at different times after grafting. Wang et al. [5] also reported significant differences in the concentrations of elements in RJ harvested at different times.

The concentrations detected in the current study were within the normal limits for most elements [23], and within the range of Mn in RJ produced in China [5]. Notably however, the Ca, Na, Mg, Fe, Zn, and Cu concentrations were higher than the ranges in RJ produced in China [5], Lithuania [34], and Bingol [9], and the concentrations of Ca, Fe, and Mn were higher than the concentrations in RJ produced in Jordan [20]. Conversely, K concentrations in the RJ samples in the current study were lower than those in RJ produced in China [5], Lithuania [34], and Bingol [9].

Concentrations of Mg, Ca, K, Na, and Mn in RJ harvested 48 hours after grafting were higher than those in RJ harvested 72 hours after grafting and 96 hours after grafting, and the lowest concentrations were detected in RJ harvested 24 hours after grafting. The high concentrations of these elements in RJ harvested at 48 and 72 hours after grafting were related to the requirements of larvae at these larval ages [8]. The respective concentrations of Mg, Ca, K, Na, Cu, and Mn in RJ harvested 48 hours after grafting were 138%, 154%, 130%, 349%, 115%, and 380% of the corresponding concentrations in RJ harvested 24 hours after grafting. In RJ harvested 72 hours after grafting the relative amounts were 132%, 130%, 121%, 331%, 114%, and 320%.

Generally, the macro elements could be arranged in a descending order: P > Mg > Ca > K > Na, and they constituted 39.8%, 34.6%, 15.2%, 8.0%, and 1.7% of the total elements quantified. Wang et al. [5] reported that K, Mg, Ca, Na, and Fe were the most abundant elements in RJ produced in China, Adaškevičiũtė et al. [34] reported that K, P, Mg, Na, and Ca were the most abundant elements in RJ from Lithuania, and Bengü et al. [9] reported that K, Mn, Mg, Ca, and Na were the most abundant elements in RJ from Bingol. Variations in macro element concentrations in RJ produced in different regions are reportedly affected by floral resources, differences in climate and geography [31, 39], and the elements in pollen consumed by nurse worker bees [40, 41].

Trace elements play a critical role in the biological characteristics of RJ due to their biological activities [9]. Fe, Zn, Cu, and Mn constituted less than 0.8% of the total estimated elements in RJ harvested at different times after grafting. Relatively similar Fe, Zn, and Cu concentrations were reportedly detected in RJ produced in China [5], Lithuania [34], and Bingol [9]. Conversely, a high concentration of Mn was reportedly detected in RJ from Bingol [9].

## Conclusions

In the current study, the concentrations of macro and trace elements in RJ differed significantly at different times after grafting. Royal jelly harvested at 48 and 72 hours after grafting had high concentrations of Mg, Ca, K, Na, Fe, Cu, and Mn and it can be used as a healthy nutritional human food supplement.
